The article "Exogenous t-PA Administration Increases Hippocampal Mature BDNF Levels. Plasmin- or NMDA-Dependent Mechanism?" was retracted in 2021. Reasons: duplicated images; original data or images not available; concerns about the data.

# Exogenous t-PA Administration Increases Hippocampal Mature BDNF Levels. Plasmin- or NMDA-Dependent Mechanism?

**DOI:** 10.1371/journal.pone.0092416

**Published:** 2014-03-26

**Authors:** Marion Rodier, Anne Prigent-Tessier, Yannick Béjot, Agnès Jacquin, Claude Mossiat, Christine Marie, Philippe Garnier

**Affiliations:** 1 Unité INSERM U1093 Cognition, Action et Plasticité Sensorimotrice, Dijon, France; 2 Université de Bourgogne, Dijon, France; 3 Département Génie Biologique, IUT, Dijon, France; 4 Department of Neurology, University Hospital, Dijon, France; 5 Centre d’Epidémiologie des Populations, EA4184, Dijon, France; Centre national de la recherche scientifique, University of Bordeaux, France

## Abstract

Brain-derived neurotrophic factor (BDNF) through TrkB activation is central for brain functioning. Since the demonstration that plasmin is able to process pro-BDNF to mature BDNF and that these two forms have opposite effects on neuronal survival and plasticity, a particular attention has been paid to the link between tissue plasminogen activator (tPA)/plasmin system and BDNF metabolism. However, t-PA via its action on different N-methyl-D-aspartate (NMDA) receptor subunits is also considered as a neuromodulator of glutamatergic transmission. In this context, the aim of our study was to investigate the effect of recombinant (r)t-PA administration on brain BDNF metabolism in rats. In the hippocampus, we found that rt-PA (10 mg/kg) administration induced a progressive increase in mature BDNF levels associated with TrkB activation. In order to delineate the mechanistic involved, plasmin activity was assessed and its inhibition was attempted using tranexamic acid (30 or 300 mg/kg, i.v.) while NMDA receptors were antagonized with MK801 (0.3 or 3 mg/kg, i.p.) in combination with rt-PA treatment. Our results showed that despite a rise in rt-PA activity, rt-PA administration failed to increase hippocampal plasmin activity suggesting that the plasminogen/plasmin system is not involved whereas MK801 abrogated the augmentation in mature BDNF levels observed after rt-PA administration. All together, our results show that rt-PA administration induces increase in hippocampal mature BDNF expression and suggests that rt-PA contributes to the control of brain BDNF synthesis through a plasmin-independent potentiation of NMDA receptors signaling.

## Introduction

Brain-derived neurotrophic factor (BDNF) serves survival and differentiation functions during the development of the nervous system [1], [2]. In addition, BDNF has been reported to be central to adult brain functions including neuronal survival, maintenance and repair, modulating dendritic branching and spine morphology [3], [4] and to be involved in activity-dependent synaptic modifications involved in learning and memory formation [5]–[7]. BDNF also represents a crucial signaling molecule in adaptative brain plasticity [8]–[10]. At the molecular level, BDNF is synthesized as pre-pro-BDNF that is processed to pro-BDNF by removal of the signal peptide. Pro-BDNF is then cleaved into mature BDNF within the endoplasmic reticulum by furin and/or in regulated secretory vesicles by protein convertase 1 whereas extracellularly, this cleavage is achieved by plasmin and some metalloproteinases [11]. Although the proteases as well as the compartment involved in the processing of pro-BDNF remain debated [12], mature BDNF signals through its high-affinity for tropomyosin-related kinase B (TrkB) receptor, thereby impacting positively brain function. Since the direct use of BDNF is limited by its pharmacokinetic profile [13], strategies aimed at inducing mature BDNF production appear to be a promising option in the treatment of variety of CNS pathologies.

Tissue plasminogen activator (t-PA) is a serine protease that has been initially characterized to promote fibrinolysis in the vascular compartment through conversion of plasminogen into plasmin. However, t-PA production is not confined to endothelial cells since it is also synthesized by neurons and glia and exerts important function in the brain parenchyma by interacting with various substrates, proteins and receptors [14], [15]. In physiological conditions, t-PA is involved during development, in neuronal migration and synaptic outgrowth while in the adult brain, t-PA is implicated in neurotransmission, synaptic plasticity and different cognitive functions [16]–[18]. However, in pathological conditions, experimental data have revealed that t-PA could have adverse effects and acts as pro-hemorrhagic and pro-excitotoxic factor [15]. To explain this multifaceted role, several plasmin-dependent and -independent mechanisms have been identified. Hence, it has been shown that t-PA through plasmin activation influences matrix degradation [19] and allows the extracellular conversion of pro-BDNF into its mature form [20], [21]. Concerning plasmin-independent mechanisms, several studies have reported in glial cells and/or in neurons that t-PA can interact with lipoprotein-receptor-related protein (LRP), annexin II and N-methyl-D-aspartate (NMDA) receptors (NMDARs) [15]. Concerning this latter, several groups have evidenced interaction and/or proteolytic implication of t-PA with different NMDAR subunits and suggested that t-PA should be also considered as a neuromodulator of glutamatergic transmission [14].

Regarding the potential link between t-PA and BDNF metabolism through either plasmin activity or activity-dependent secretion of BDNF through elevation of intracellular calcium levels mediated by the activation of NMDA receptors, the objective of our study was to investigate the effect of exogenous t-PA administration (recombinant (r)t-PA) on brain levels of mature BDNF in rats. In order to gain insight into mechanistic, rt-PA and plasmin activities were measured and a pharmacological approach using non-subunit-specific MK801 targeting NMDARs and tranexamic acid (TXA) as plasmin inhibitor was designed. In addition, the activation of TrkB receptors was assessed.

## Materials and Methods

### Reagents

Acrylamide and bis-acrylamide, sodium dodecylsulfate (SDS) and tween-20 were obtained from Bio-Rad (Ivry sur Seine, France). The polyvinylidene difluoride (PVDF) membranes were purchased from GE Healthcare (Orsay, France). For Western blotting assessments, rabbit polyclonal anti-pro-BDNF (AB5613P) antibody was obtained from Merck-Millipore whereas the rabbit monoclonal antibody recognizing both BDNF forms (clone EPR 1292, Ref. 3160-1) was purchased from Epitomics (Euromedex, Souffelweyersheim, France). The mouse monoclonal antibody raised against TrkB full length (ref 610102) and the rabbit polyclonal recognizing TrkB phosphorylated at tyrosine 515 (ab51187) were obtained from BD Biosciences (Franklin Lakes, US) and Abcam (Cambridge, UK), respectively. Mouse monoclonal anti-β-actin antibody (A5441) was purchased from Sigma-Aldrich (St Louis, MO). For secondary antibodies, the horseradish peroxidase-conjugated anti-rabbit and -mouse antibodies were obtained from Jackson ImmunoResearch Laboratories (Interchim, France). For pharmacological approaches, rt-PA (Actilyse), tranexamic acid (Exacyl) were purchased from Boehringer Ingelheim (Paris, France) and Sanofi Aventis (Paris, France) whereas MK801 (Ab120027) was obtained from Abcam (Cambridge, UK).

### Animals

The experiments were carried out on adult male Wistar rats (290–310 g; Depré, Saint-Doulchard, France) and were conducted according to the French Department of Agriculture guidelines (license 21CAE099) and performed in order to comply with the ‘*Animal Research: Reporting In Vivo Experiments*’ ARRIVE guidelines. The animals were housed five per cage and kept under 12/12 h light/dark cycle and allowed *ad libitum* access to food and water. The experimental procedures were approved by the local committee for ethic in animal experimentation (agreement 6112). All efforts were made to minimize animal suffering and to reduce the number of animals used. Due to the duration of anesthesia and the potential effects of barbiturate [22] and ketamine [23] on NMDA receptor signaling, all surgery was performed under chloral hydrate anesthesia (400 mg/kg, i.p.). Head/body temperatures were monitored and controlled during surgical procedure. The choice of doses and the route of administration of drugs have been made in agreement with the literature. All treated animals have been included in this study. In order to minimize the impact of circadian cycle, animals were homogeneously allocated in each group with respect to the time of day at which the injection occurred.

After anesthesia (400 mg/kg; chloral hydrate; i.p.), animals were perfused with vehicle (L-Arginin 3.5% in deionized water, n = 10) or rt-PA 10 mg/kg i.v. (undialyzed, n = 10) combined or not with tranexamic acid (30 or 300 mg/kg, n = 5 and n = 8, respectively) as a bolus (10% of total dose) followed by a 60 min perfusion (90% of total dose) using pump infusion (Harvard Apparatus, 55–4150) to mimic the clinical utilization of rt-PA. For MK801 treatments, two doses were used (0.3 or 3 mg/kg, i.p., n = 5 and n = 8, respectively) as a bolus immediately after the beginning of vehicle or rt-PA infusion. Since blood contains BDNF, 2 h or 24 h after the beginning of drugs administration, animals were transcardially perfused with saline during 5 min to flush out blood from vasculature to avoid contamination, and then, the brains were removed. The cortices, striatum and hippocampi were quickly dissected on glass slide at 0°C. The different brain structures were immediately weighted and frozen at −80°C until further use.

### Western Blotting

To assess the expression of the pro-BDNF, mature BDNF, Full length (FL)-TrkB, phosphorylated (p)-TrkB and β-actin by Western blotting analyses, the different cerebral samples were first homogenized in seven volumes of lysis buffer [bi-distilled water containing 100 mM Tris, 150 mM NaCl, 1 mM EGTA, 1% triton X-100, 1% protease inhibitors (Sigma P8340)] as previously described [24]. Then, the total protein extracts were sonicated and centrifuged at 14,000×*g* for 20 min. An aliquot of supernatant was kept for BCA protein measurement and the remaining protein extracts were stored at −80°C.

Equal amounts of proteins were dissolved in Laemmli solution (62.5 mM Tris–HCl (pH 6.8), 2% SDS, 10% glycerol, 0.001% bromophenol blue) with 2-mercaptoethanol 5% and were heated at 85°C for 10 min. Proteins were separated on 10% (p-TrkB) or 12% (Pro-BDNF, FL-TrkB and mature BDNF) SDS–polyacrylamide gel electrophoresis (PAGE) and were electrophoretically transferred onto PVDF membrane (0.2 μm pore size) in cold transfer buffer [10 mM NaHCO_3_, 3 mM Na_2_CO_3_ (pH 9.9) and 20% methanol]. Specificity of the different BDNF antibodies was characterized previously [25]. The membranes were incubated overnight at 4°C in 5% non-fat dry milk or 7.5% BSA (p-TrkB) in TBS [20 mM Tris–HCl (pH 7.6) and 137 mM NaCl] containing 0.1% Tween 20 to block unspecific binding. They were then washed, incubated for 3 h at room temperature (RT) with anti-pro-BDNF (1/2000), anti-BDNF (1/3000 with 5% non fat dry milk), anti-FL-TrkB (1/1000), anti p-TrkB (1/1000 with 5% BSA) or anti-β-actin antibodies (1/5000). The membranes were washed with TBS-0.1% Tween 20 and then incubated for 2 h (RT) with either horseradish peroxidase (HRP)-conjugated anti-mouse IgGs or anti-rabbit IgGs. Protein-antibody complexes were visualized using enhanced chemiluminescence Western blotting detection system according to the manufacturer’s protocol (ECL+, GE Healthcare, Orsay, France). The membranes were stripped and probed with an anti-β-actin antibody (1/5000) used as internal control. Pro- and mature BDNF, FL-TrkB, p-TrkB and β-actin band densities were determined by scanning densitometry (GS-800, Bio-rad, Ivry sur Seine, France). A computer-based imaging system (Quantity One, Bio-rad, Ivry sur Seine, France) was used to measure the relative optical density of each specific band. Data normalized on β-actin expression were expressed as percentage of increase as compared to control values.

### t-PA Activity Assay

t-PA activity was measured using Sensolyte AMC t-PA Activity Assay (Anaspec, TEBU Bio, Le Perray-en-Yvelines, France) according to the manufacturer’s protocol. Of note, measurements were performed on brain homogenates prepared as previously described for Western blotting experiments without protease inhibitors. Briefly, 50 μl of fluorimetric substrate was incubated with 50 μl of the different brain extracts. Measurements were performed in duplicate at 30°C over a 60 min period using multiplate reader (Wallac Victor^2^ 1420 Multilabel Counter). Relative fluorescent unit (RFU) per min were normalized by protein concentration and data were expressed as percentage of increase as compared to control values.

### Plasmin Activity Assay

Plasmin activity was measured using Sensolyte Rh 110 Plasmin Activity Assay (Anaspec, TEBU Bio, Le Perray-en-Yvelines, France) according to the manufacturer’s protocol. Measurements were performed on brain homogenates prepared as previously described for Western blotting experiments without protease inhibitors. Briefly, 50 μl of fluorimetric substrate was incubated with 100 μl of the different brain extracts and 50 μl of serum diluted to one-tenth in saline. Measurements were performed in duplicate at 30°C over a 60 min period using multiplate reader (Wallac Victor^2^ 1420 Multilabel Counter). Relative fluorescent unit (RFU) per min were normalized by protein concentration and data were expressed as percentage of increase as compared to control values.

### Statistics

All values were expressed as means ± S.E.M. of n rats (five to ten animals in each group). Comparisons among groups of rats were made using non-parametric Kruskal–Wallis test followed by Mann–Whitney for independent variables. All statistical analysis was performed using systat 9.0 software (SPSS Science SoftwareGmb, Erkrath, Germany). Statistical significance was set at P<0.05.

## Results

### Effect of rt-PA on t-PA Activity and Mature BDNF Expression

t-PA activity and mature BDNF expression were assessed in the striatum, the cortex and the hippocampus 2 h and 24 h after administration of either rt-PA (10 mg/kg, i.v., n = 10) or vehicle (n = 10). Concerning t-PA activity (figure 1), our results revealed that rt-PA induced a significant increase only in the hippocampus, 2 h and 24 h after perfusion as compared to vehicle treated animals. Concerning mature BDNF expression, Western blotting assessments showed that rt-PA treatment was associated with a significant and progressive rise of mature BDNF only in the hippocampus (Figure 2). Regarding both t-PA activity and mature BDNF expression in other brain regions, rt-PA exerted no significant effect and thus, whatever the time points considered.

**Figure 1:** Effect of rt-PA (10 mg/kg) on t-PA activity in different brain structures. t-PA activity was assessed 2 h and 24 h after rt-PA or vehicle perfusion in the striatum, cortex and hippocampus. Data are presented as mean ± SEM and are representative of 10 animals. *P<0.05 and **P<0.01 compared to vehicle-treated animals.

**Figure 2:** mature BDNF expression in different brain structures. Mature BDNF (mBDNF) expression was assessed 2 h and 24 h after rt-PA or vehicle perfusion in the striatum, cortex and hippocampus. Representative immunoblots are shown and densitometric analysis was performed after normalization of mBDNF expression on β-actin levels. Data are presented as mean ± SEM and are representative of 10 animals. *P<0.05 and **P<0.01 compared to vehicle-treated animals.

### Effect of TXA on rt-PA-induced Mature BDNF Expression

In order to evaluate the involvement of plasmin on rt-PA-induced mature BDNF upregulation in the hippocampus, animals received rt-PA perfusion combined with TXA (30 or 300 mg/kg, i.v.). As compared to animals treated with rt-PA alone (n = 10) (Figure 3A), no significant differences were observed in animals treated with rt-PA and TXA at either 30 or 300 mg/kg (n = 5 and n = 8, respectively). Indeed, animals treated with both pharmacological agents showed a significant increase in mature BDNF expression. Of note, animals treated with TXA alone, showed no variation in mature BDNF expression as compared to vehicle-treated animals (data not shown).

**Figure 3:** Effect of tranexamic acid on rt-PA-induced increase in mature (A) and proBDNF (B) expressions in the hippocampus. Animals received rt-PA or vehicle perfusion associated or not with tranexamic acid (TXA) (30 or 300 mg/kg). Western blotting assessments were performed 2 h and 24 h after administration of the different treatments. Representative immunoblots are shown and densitometric analysis was performed after normalization of mature BDNF (mBDNF) and proBDNF expressions on β-actin levels. Data are presented as mean ± SEM and are representative of 5 to 10 animals. *P<0.05 and **P<0.01 compared to vehicle-treated animals.

### Effect of rt-PA and TXA on Plasmin Activity

Plasmin activity was performed in the hippocampus 2 h after administration of rt-PA (10 mg/kg, i.v., n = 7), TXA (300 mg/kg, n = 7), rt-PA in combination with TXA (n = 7) or vehicle (n = 7). Plasmin activity in the serum of animals treated by rt-PA was also assessed and used as a positive control. As compared to the major increase in plasmin activity measured in the serum of rt-PA treated animals (+1500%), no variation was detected in the hippocampic homogenates of rats treated either by rt-PA, TXA alone or rt-PA and TXA acid (Figure 4). Of note, plasmin activity in vehicle-treated animals was found very low, barely detectable in the hippocampal tissue as compared to the circulating compartment (1.3 RFU/min/μg vs 12.2 RFU/min/μg, respectively).

**Figure 4:** Effect of rt-PA (10 mg/kg) associated or not with tranexamic acid (TXA, 300 mg/kg) on plasmin activity in the serum and the hippocampus. Plasmin activity was assessed 2-PA perfusion in the serum and 2 h after vehicle, t-PA alone or in association with TXA and TXA alone in the hippocampus. Data are presented as mean ± SEM and are representative of 7 animals. **P<0.01 compared to vehicle-treated animals.

### Effect of MK801 on rt-PA-induced Mature BDNF Expression

To assess whether the increase in hippocampal mature BDNF expression induced by rt-PA could be mediated by the potentiation of NMDA receptor signaling, animals received rt-PA in association with MK801 (0.3 or 3 mg/kg, i.p., n = 5 and n = 8, respectively). Our data revealed that MK801 combined with rt-PA abolished the increase in mature BDNF expression induced by rt-PA administration (Figure 5A), This abrogation was observed at both doses of MK801. Of note, animals treated with MK801 alone, showed no difference in term of mature BDNF expression as compared to vehicle-treated animals (data not shown).

**Figure 5:** Effect of MK801 on rt-PA-induced increase in mature (A) and proBDNF (B) expressions in the hippocampus. Animals received rt-PA or vehicle perfusion associated or not with MK801 (0.3 or 3 mg/kg). Western blotting assessments were performed 2 h and 24 h after administration of the different treatments. Representative immunoblots are shown and densitometric analysis was performed after normalization of mature BDNF (mBDNF) and proBDNF expressions on β-actin levels. Data are presented as mean ± SEM and are representative of 5 to 10 animals. *P<0.05 and **P<0.01 compared to vehicle-treated animals.

### Effect of rt-PA alone or in Association with TXA or MK801 on Pro-BDNF Expression

In order to assess whether rt-PA-induced mature BDNF expression was associated with variations in pro-BDNF expression, Western blotting assessments were performed 2 h and 24 h after drugs administration in the hippocampus. Our results showed that rt-PA alone (Figure 3B and 5B) or in combination with TXA (Figure 3B) or with MK801 (Figure 5B) induced no significant change in pro-BDNF expression as compared to vehicle-treated animals. In addition, TXA or MK801 alone induced no variation in pro-BDNF expression as compared to vehicle-treated animals (data not shown).

### Effect of rt-PA alone or in Association with TXA or MK801 on TrkB Receptor Activation

To evaluate whether changes in mature BDNF expression paralleled with changes in TrkB receptor activation, we measured the impact of rt-PA alone or combined with tranexamic acid or MK801 on the ratio of p-TrkB to FL-TrkB levels (Figure 6). Our results showed that the conditions inducing an increase in mature BDNF expression at both 2 h and 24 h were associated with a significant elevation of the p-TrkB/FL-TrkB ratio at 24 h. Indeed, rt-PA-treated animals (n = 10) and rt-PA-TXA-treated (30 mg/kg, n = 5 and 300 mg/kg, n = 8) animals exhibited a significant increase in this ratio as compared to vehicle-treated animals. However, our data revealed that when co-treated with MK801, rt-PA-treated animals showed no longer increase in the p-TrkB/FL-TrkB ratio. Of note, MK801 and TXA alone (both doses) induced no change in the p-TrkB/FL-TrkB ratio (data not shown).

**Figure 6:** Effect of rt-PA (10 mg/kg) associated or not with tranexamic acid or MK801 on the ratio p-TrKB/FL-TrKB expression. Western blotting assessments were performed 2-TrkB and FL-TrkB expressions on β-actin levels. Data are presented as mean ± SEM and are representative of 5 to 10 animals. *P<0.05 compared to vehicle-treated animals. NS = non-significant.

## Discussion

Regarding the relevance of stimulating BDNF metabolism in various CNS pathologies [26], [27], the objective of our study was to assess the effect of exogenous t-PA administration in the maturation of this neurotrophin. For this purpose, we studied the effect of rt-PA on the expression of both pro-BDNF and its mature form and we delineate the mechanistic involved through a pharmacological approach. The present study reveals that i) rt-PA induced a rise in mature BDNF expression and subsequent TrkB receptor activation and that these effects are ii) region-dependent and iii) mediated by NMDAR activation rather than through increase in plasmin activity.

Since the initial *in vitro* demonstration that proteolytic conversion of pro-BDNF to mature BDNF can be achieved by extracellular proteases such as the t-PA/plasmin system [20], [28] and that these two BDNF forms have the propensity to produce diametrically opposite effects on neuronal survival and plasticity [11], a particular attention has been paid to the potential relation between t-PA activity and BDNF metabolism. *In vivo*, endogenous brain t-PA activity has been shown to be increased by enriched environment [29], [30], electroconvulsive therapy [31] and after physical activity paradigms [32] whereas prenatal restraint stress of rat dams induces decrease in t-PA activity in the offspring of both sexes [33]. Interestingly, a positive link has been established between t-PA activity and mature BDNF levels in these studies, suggesting the implication of t-PA in the maturation of BDNF. Using systemic administration of rt-PA as an original approach to increase t-PA activity, the present study provides strong arguments for the contribution of t-PA-dependent mechanism in the control of mature BDNF expression. Of note, our results showed that t-PA administration increased significantly t-PA activity only in the hippocampus. Since it has been shown that blood-brain barrier is permeable to t-PA [34] and reported that endogenous content of t-PA inhibitors differ among the different brain structures [35], our data suggest a low level of these inhibitors in the hippocampus.

Recent literature reports that t-PA could act on BDNF metabolism through a plasmin-dependent processing of pro-BDNF to the mature form. Although debated [12], these assertions came initially from *in vitro* studies using neuronal culture. Hence, it has been shown that upon high frequency stimulation, the extracellular cleavage of pro-BDNF was reduced when cultured hippocampal neurons were treated with the membrane impermeable plasminogen activator inhibitor-1 [21]. More recently, the implication of t-PA/plasmin system was also suggested *in vivo*, in studies showing that physical exercise induces a correlation between mature BDNF levels and t-PA gene induction [36] and more strikingly, that 2,7-Bis-(4-Amidinobenzylidene)-Cycloheptan-1-one Dihydrochloride (t-PA STOP) blocks exercise-induced increase in mature BDNF expression [32]. In order to assess whether plasmin activation was implicated in the increase in mature BDNF expression observed in rt-PA-treated animals, we modulated plasmin activity through tranexamic acid, a synthetic lysine analog that shows high affinity to lysine binding sites of plasminogen and plasmin. Using two different doses, when injected in combination with rt-PA, tranexamic acid failed to counteract the rise in mature BDNF expression observed in animals receiving rt-PA alone. Although tranexamic acid induces convulsions in animals [37] and is contraindicated in epileptic patients, the absence of direct arguments for the penetration of this compound from blood to brain could explained this observed lack of effects. In order to clarify these data, we measured through specific enzymatic assay, hippocampal plasmin activity in control animals and in animals treated by rt-PA alone or in association with tranexamic acid. As compared to vehicle-treated animals, rt-PA induced no increase in plasmin activity in the hippocampal tissues despite a major rise in the circulating compartment. In addition, in the hippocampal area, basal plasmin activity was found barely detectable suggesting that plasmin activity is locally controlled to avoid a deleterious extracellular proteolysis. In line with this assumption, several studies have reported that the principal physiological plasmin inhibitor, the α2-antiplasmin, is highly expressed in rodent hippocampus [38], [39]. Besides, it has been shown that the t-PA substrate plasminogen is localized intracellularly, mainly in the neuronal somata of the CA3 and CA1 layers [40]. Overall data suggest that rt-PA-induced increase in hippocampal mature BDNF expression is a plasmin-independent mechanism.

As stated in the introduction, t-PA effect is not restricted to plasmin-dependent mechanisms. Among its different functions, t-PA is now considered as a neuromodulator of glutamatergic signaling mediated by NMDARs. Indeed, t-PA has been shown to interact with NMDAR subunits such as GluN1, GluN2B and GluN2D with several potential mechanisms [14], [15]. Thus, it has been reported that t-PA could increase NMDAR calcium permeability through proteolytic cleavage of the amino terminal domain of the GluN1 subunit [41], [42]. In addition, the interaction between t-PA and GluN2B subunit has been reported in the setting of alcoholism leading to an upregulation of GluN2B-containing NMDA receptors [43] while more recently, a preferential activation with GluN2D subunit-containing NMDA receptors influencing spatial memory has also been evidenced [44]. Besides, t-PA might modulate indirectly NMDA-evoked current through its ability to signal via LRP-1, a membrane receptor tethered to NMDARs by the intracellular scaffold protein, PSD-95 [45]. Regarding the potential multi-subunit interactions of t-PA with NMDAR, we choose the non-subunit-specific NMDAR antagonist MK-801 to assess whether the increase in mature BDNF expression observed in rt-PA-treated animals could be mediated by NMDAR activation. When injected just after the beginning of rt-PA perfusion, both doses of MK801 completely negated the rise in mature BDNF expression induced by rt-PA, strongly suggesting that the increase in hippocampal mature BDNF expression is mediated by a rt-PA impact on NMDAR signaling. Regarding the mechanism potentially involved, it can be suggested that calcium influx induced by NMDAR activation could induce BDNF gene expression as suggested by a study showing in rats that exercise-induced increase in hippocampal BDNF mRNA levels is completely prevented by NMDAR blockade [46] and/or that NMDAR activation could impinge activity-dependent secretion of mature BDNF [47]. According to the evolution of pro-BDNF expression that was found stable over the different time points despite an increase in the mature form, our data could support the idea that rt-PA-induced increase in mature BDNF expression results from the processing of pro-BDNF associated with its continuous synthesis. In addition, although the precise interactions of rt-PA with the different NMDAR subunits are not investigated here, it is conceivable to hypothesize that the confinement of rt-PA-induced increase in mature BDNF expression to the hippocampus could be due to the specific composition in NMDAR subunits of this brain structure [48], [49]. This hypothesis is in line with a study showing that rt-PA incubation increased survival in hippocampal but not in cortical neurons exposed to oxygen-glucose deprivation [50]. Finally, as compared to *in vivo* studies concluding on the involvement of the t-PA/plasmin by showing that t-PA STOP blocked exercise-induced mature BDNF expression [32], our results could lead to a reinterpretation. Indeed, it is important to notice that t-PA STOP has also been shown to attenuate t-PA-dependent potentiation of NMDA-induced calcium influx [51].

By virtue of its essential role in development, neuronal health and plasticity, BDNF deregulation has been implicated in many psychiatric disorders [27]. In addition, regarding its contribution to post-stroke neuroplastic changes [8], [10], strategies aiming at upregulating mature BDNF levels or mimicking BDNF signaling may offer clinically relevant therapeutics. In the present study, we also analyzed whether the rise in mature BDNF observed in rt-PA-treated animals was associated with the activation of its high affinity receptor TrkB by assessing the phosphorylation state of this receptor. Our data revealed that the increase in mature BDNF levels after rt-PA treatment was associated with TrkB receptor activation. In addition, a causative link between mature BDNF expression and TrkB receptor phosphorylation was suggested since MK801 but not tranexamic acid, abolished TrkB receptor activation. According to the fact that BDNF binding to TrkB receptors elicits several intracellular signaling cascades that mainly impact neuronal outcome positively [52], t-PA administration or interventions aimed at increasing t-PA activity such as physical exercice [32] could represent an interesting strategy in various neurological and psychiatric disorders associated with low level of BDNF and/or requiring an overproduction of this neurotrophin. Besides, since rt-PA-induced increase in mature BDNF and subsequent TrkB receptor activation occurred only in the hippocampus, it can be hypothesized that exogenous t-PA could impact activity-dependent synaptic modifications and induce neurogenesis and improve memory formation in this structure. Lastly, strategies aimed at increasing t-PA activity could be specially relevant in humans carrying val66met polymorphism that are suspected to have a reduced activity-dependent BDNF secretion and are subjected to impaired episodic memory function [27] and are at risk for psychiatric diseases [53].

In conclusion, the present study strongly suggests that exogenous t-PA induces increase in hippocampal mature BDNF expression through NMDAR activation. Although our results do not presage the mechanisms that would be implicated in pathophysiological situations such as stroke in which t-PA has also been reported to potentiate NMDAR signaling to an excitotoxic threshold [48], [54], overall results may underlie a possible beneficial, structure-dependent and extra-fibrinolytic effect of exogenous t-PA. Since rt-PA is the only approved treatment of thromboembolic stroke, the potential occurrence of similar mechanisms in experimental stroke models warrants future studies.
